The article "The Efficacy and Safety of Anlotinib Alone and in Combination with Other Drugs in Advanced Lung Cancer: A Retrospective Cohort Study" was retracted in 2023. Reasons: signs of a paper mill; suspected computer-generated content; unreliable results or conclusions; concerns about the data.

# The Efficacy and Safety of Anlotinib Alone and in Combination with Other Drugs in Advanced Lung Cancer: A Retrospective Cohort Study

**DOI:** 10.1155/2022/1475871

**Published:** 2022-02-25

**Authors:** Lei Li, Hui Zhang, Yalin Xie, Ning Su, Shan Su, Xianlan Zhang, Wenchang Cen

**Affiliations:** Department of Oncology, Guangzhou Chest Hospital, Guangzhou, China

## Abstract

**Objective:**

Lung cancer is a disease associated with high levels of morbidity and mortality, with approximately 2.1 million new cases every year. Anlotinib is a new small-molecule multitarget tyrosine kinase inhibitor independently developed in China that can inhibit the formation of tumor blood vessels and has a therapeutic effect on various cancers. However, the application of anlotinib in lung cancer needs further investigation.

**Methods:**

We collected the progress notes of 43 patients with advanced lung cancer treated at the Oncology Department of Guangzhou Chest Hospital from March 2019 to March 2021. Additionally, we assessed the differences between drug combination therapy and single-drug therapy among patients treated with anlotinib.

**Results:**

Patients in both the anlotinib-combination and anlotinib-monotherapy groups experienced remission; however, the overall disease control rate in the anlotinib-combination group was higher than that in the anlotinib-monotherapy group. Reexamination via computed tomography showed that patients in the anlotinib-combination group had better recovery than those in the anlotinib-monotherapy group. Although the overall incidence of adverse reactions in the anlotinib-combination group was higher than that in the monotherapy group, most of the adverse reactions were I–II levels and improved after symptomatic treatment.

**Conclusion:**

Anlotinib combined with other therapies is better than anlotinib alone for the management of patients with advanced lung cancer.

## 1. Introduction

Lung cancer is the primary cause of death due to malignancies worldwide and is associated with high morbidity and mortality. There are approximately 2.1 million new cases and 1.77 million new deaths worldwide annually, and lung cancer poses a serious threat to people's life, health, and safety [1, 2]. Lung cancer is classified as either non-small-cell lung cancer (NSCLC) or SCLC based on pathological tissue types; among these, NSCLC is the most common. The disease in most patients with NSCLC appears to have progressed to the middle and terminal stages at the time of diagnosis, leading to patients missing the optimal period for surgery [3]. Moreover, NSCLC has a 5-year survival rate of less than 15% [4, 5]. Therefore, chemotherapy is the primary treatment for these patients. Targeted treatment and immunotherapy have improved progression-free survival (PFS) and overall survival (OS) in patients with NSCLC [6, 7].

Many scholars have found that lung cancer develops due to activating mutations of many driver genes, such as epidermal growth factor receptor (EGFR), anaplastic lymphoma kinase (ALK), c-ROS oncogene 1 receptor tyrosine kinase (ROS1), and Kirsten rat sarcoma viral oncogene [8, 9]. The discovery of these mutated genes has spurred many new research directions for targeted therapy for NSCLC. Targeted therapy for some genes has been widely successful [10]. For example, crizotinib, the first ALK inhibitor, reduces ALK activity by inhibiting the binding of ALK to ATP and its own phosphorylation after binding. Clinical studies have shown that crizotinib is significantly better than traditional chemotherapy in the treatment of PFS for lung adenocarcinoma [11]. Entrectinib is a novel ROS1, tropomyosin receptor kinase, and ALK combined inhibitor, which affects a variety of solid tumor cells. Studies have shown that the median PFS of ROS1-positive patients is relatively prolonged after treatment with entrectinib [12].

Despite great development in targeted therapy and immunotherapy in the past decade, patients with NSCLC do not respond well in the presence of treatment resistance [13]. Studies have shown that the proliferation of cancer cells requires the establishment of new blood vessels to obtain energy, and the cell signal transduction mediated by vascular endothelial growth factor and its receptor, vascular endothelial growth factor receptor (VEGFR), is involved in and regulates tumor angiogenesis [14, 15]. Clinically, there are EGFR–tyrosine kinase inhibitor-targeted therapies for EGFR, which can inhibit tyrosine kinase, inhibit epidermal growth factor upregulation, or delay and inhibit tumor invasion or metastasis, and these therapies have been proven to be effective in the treatment of NSCLC [16].

Anlotinib is a novel small-molecule multitarget tyrosine kinase inhibitor independently developed in China, and it mainly inhibits VEGFR, fibroblast growth factor receptor, platelet-derived growth factor, and stem cell factor receptor. It also controls tumor growth and plays an antitumor role in VEGFR to inhibit tumor angiogenesis [17]. In May 2018, anlotinib was approved by the China Food and Drug Administration for the third-line treatment of patients with advanced NSCLC [18]. This study is aimed at retrospectively analyzing the safety and efficacy of anlotinib combined with other treatment regimens in patients with advanced stages of cancer to provide evidence on the third-line and above clinical treatment.

## 2. Methods

### 2.1. Patient Selection

Data on the 43 patients in this study were collected from those admitted to Guangzhou Chest Hospital from March 2019 to March 2021. Patients presented for medical treatment due to discomfort and underwent pathological examination, computed tomography (CT), or magnetic resonance imaging during the outpatient or hospital stay. An example of a patient's CT is shown in Figure 1; the image shows spinous nodules in the left lung and local lung tissue calcification. Ultimately, the doctor diagnosed lung cancer, and based on this diagnosis, the doctor prescribed treatment with anlotinib. All patients provided signed informed consent before medication, and all had advanced lung cancer requiring second-line treatment or above. The patients had comorbidities, including essential hypertension, diabetes, coronary heart disease, tuberculosis, and pulmonary bullae. All patients took oral medications, and their conditions were stable. The study was approved by the Ethics Committee of Guangzhou Chest Hospital. Informed consent was obtained from the participants prior to enrollment in the study.

### 2.2. Treatment and Follow-Up

According to the treatment plan, patients were divided into 2 groups: anlotinib-monotherapy (17 patients) and anlotinib-combination therapy (26 patients), as shown in Figure 2. All included patients met the following criteria: (1) an Eastern Cooperative Oncology Group (ECOG) scores 0–3; (2) diagnosed based on pathological examination; (3) CT or magnetic resonance imaging could be used to measure the lesion; (4) blood routine, blood coagulation, and liver and kidney function were normal; and (5) expected survival duration was longer than 3 months. Patients with the following were excluded: (1) hemoptysis, hematemesis, or hematochezia; (2) uncontrollable hypertension or proteinuria; and (3) other uncontrollable factors or refusal to receive treatment.

All patients were administered anlotinib hydrochloride 12 mg daily for 2 weeks followed by cessation for 1 week. The anlotinib-combination group (combination chemotherapy, immunotherapy, or molecular targeted therapy) was treated with anlotinib in combination with osimertinib, sintilimab, tegafur gimeracil, and oteracil potassium or chemotherapy. All patients' blood parameters, urine parameters, and liver and kidney function were regularly checked every 3 weeks. If a patient developed severe grade V hypertension, hand-foot syndrome, proteinuria, hematologic adverse reactions, or combined infections, and the patient was intolerant, the dose of anlotinib hydrochloride was reduced to 10 mg/day, or the medication was discontinued. A total of 21 days comprised 1 cycle, and 1 cycle of treatment was used to evaluate the efficacy and adverse reactions. The treatment lasted for 4 cycles.

### 2.3. Statistical Analysis

Data were analyzed using the GraphPad Prism 9.1 statistical software. Continuous variables were expressed as mean ± standard deviation (SD). Chi-squared or Fisher's exact tests were used for analyzing differences between the groups. A value of *P* < 0.05 was considered statistically significant.

## 3. Results

Patient data are shown in Table 1. On comparison of the anlotinib-monotherapy group with the anlotinib-combination group, no significant differences in the proportion of men and women, age range, or ECOG score between the 2 groups (*P* > 0.05) were observed. A total of 33 patients received tumor cell genetic testing; 19 had an EGFR mutation (19del, 20ins 21L858R), 9 had the ALK fusion gene, 9 had a ROS1 gene mutation, and 3 had a HER2 mutation. There were significant differences in the type of gene mutation and smoking between the 2 groups (*P* < 0.05). Therefore, the mutation of specific genes may have a certain influence on the choice of treatment plan.

### 3.1. The Effectiveness of Treatment

After 1 cycle of treatment, the Response Evaluation Criteria in Solid Tumors was used to evaluate the short-term efficacy in each group. The results are shown in Table 2. Overall, there were 7 cases of PR, 22 cases of SD, and 14 cases of PD among the patients with lung cancer. The overall remission rate (ORR) and disease control rate (DCR) were 16.28% (7/43) and 67.44% (29/43), respectively. In terms of ORR and DCR, the rates were lower in the anlotinib-monotherapy group than in the anlotinib-combination group, and the differences were statistically significant (*P* < 0.05). Therefore, anlotinib-combination therapy may be more effective in the treatment of advanced lung cancer than anlotinib alone.

After several months of treatment, patients in both the groups were examined using CT. As shown in Figure 3, the treatment results indicated that the ground glass shadow of the right lung did not change significantly in the patients treated with anlotinib, and the white mass area of the left lung had decreased slightly, showing no obvious therapeutic effect.  Figure 4 shows that the right lower lung mass shadow and consolidation shadow disappeared in the anlotinib-combination group, and the right lung tissue returned to normal, showing an obvious treatment effect.

### 3.2. Adverse Reaction Analysis

During the treatment, hypertension, rash, diarrhea, nausea and vomiting, leukopenia, decreased appetite, and anemia occurred in both the groups, all of which improved after symptomatic treatment. Most of the reactions were grades I and II (Table 3). One patient in the anlotinib-monotherapy group had a dose of anlotinib hydrochloride decreased from 12 mg/d to 10 mg/d due to grade III proteinuria. One patient in the combination group discontinued anlotinib hydrochloride due to grade III creatinine elevation, and none of the remaining patients adjusted their dose. The incidences of hypertension, proteinuria, nausea and vomiting, creatinine increase, and other adverse reactions in the anlotinib-monotherapy group were lower than those in the anlotinib-combination group; the difference was statistically significant (*P* < 0.05). All data were followed up until March 1, 2021, for a period of 1–20 months.

## 4. Discussion

Patients with advanced NSCLC have a shorter survival, with a 5-year OS of less than 5%. First- and second-line treatment options include chemotherapy, targeted therapy, and immunotherapy [19, 20]. However, due to the occurrence of adverse drug reactions and drug resistance as well as the high price of immunotherapy, new options need to be explored [21]. At present, the standard first-line chemotherapy is the platinum-based 2-drug regimen; however, the adverse drug reactions are relatively serious, the efficacy is difficult to improve, and patients who fail multiline chemotherapy have less chances of benefiting from chemotherapy [22].

As a new class I drug developed by China with independent intellectual property rights, anlotinib has achieved effective third-line treatment for advanced or metastatic NSCLC. It provides a new drug choice for patients with cancer to relieve pain, prolong life, and improve the quality of life [23].

In this study, anlotinib alone or in combination with other therapeutic methods was used to explore the most effective treatment method employing anlotinib. There were significant differences in EGFR mutations and the number of smokers between the two treatment regimen groups, suggesting that mutations and smoking could affect the treatment regimens. In clinical practice, genetic testing has become an important means of cancer diagnosis [24]. EGFR, BRAF, and MET mutation detection have even been included in the diagnostic criteria of NSCLC [25, 26]. Drugs targeting these mutated genes have been used in clinical setting with good efficacy. Combined with this data analysis, given that patients in the combination therapy group had more types of gene mutations, the corresponding targeted therapy was preferred in clinical practice.

According to ORR and DCR statistics, anlotinib combined with other therapeutic methods can effectively control and alleviate lung cancer, and the disease control efficiency is better than that of anlotinib-monotherapy. The patients' CT results also showed that anlotinib-combination therapy was more effective for lung cancer, and that patients recovered faster. The incidences of hypertension, proteinuria, nausea and vomiting, and increased creatinine were higher in the combination group; however, most of them were grade I and II reactions that improved after symptomatic treatment. This result shows that anlotinib combined with other treatments has better therapeutic effect and safety than anlotinib alone.

This study has some limitations. Due to insufficient experimental data, patient survival analysis could not be conducted, and the efficacy analysis of anlotinib treatment is insufficient. More cases should be analyzed, and anlotinib patient survival should be studied separately.

In conclusion, for the third-line treatment of patients with advanced lung cancer, anlotinib, combined with other treatment methods, has a good effect on the disease control and patients' remission rates. Anlotinib is effective for the treatment of advanced lung cancer.

## Figures and Tables

**Figure 1:** Computed tomography-based diagnosis of lung cancer in a patient. (a) Coronal reconstruction. (b) An axial scan.

**Figure 2:** Experimental group flow chart.

**Figure 3:** CT images of the lungs of patients in the anlotinib group showed a large area of ground glass shadow in the right lower lung. (a) Patients before treatment. (b) Patients after treatment. The left side shows a coronal reconstruction, and the right shows an axial scan.

**Figure 4:** CT images of the patients in the anlotinib-combination group; the right lower lung mass shadow disappeared after treatment. (a) Patients before treatment. (b) Patients after treatment. The left side shows a coronal reconstruction, and the right shows an axial scan.

**Table 1:** Analysis of patients' basic data.

Clinical bed characteristics	Anlotinib (*n* = 17)	Combination (*n* = 26)	*P*
Gender			0.362
Male	10	17	
Female	7	9	
Age			0.739
≥60	8	16	
<60	9	10	
ECOG score			0.429
0-1	14	20	
≥2	3	6	
Smoking status			0.037^∗^
Smoker	6	12	
Nonsmoker	11	14	
Histology			0.581
Adenocarcinoma	11	17	
Squamous cell carcinoma	4	6	
Other types	3	2	
Genetic testing (*n* = 33)			0.043^∗^
EGFR mutation	7	12	
HER2 mutation	2	1	
Other types	3	8	

Compared with the anlotinib group, ^∗^*P* < 0.05.

**Table 2:** Comparison of short-term efficacy between the anlotinib-monotherapy group and the anlotinib-combination group.

	*n*	CR	PR	SD	PD	ORR	DCR
Anlotinib	17	0	2	8	7	2 (11.8%)	10 (58.8%)
Combination therapy	26	0	5	14	7	5 (19.2%)	19 (73.0%)
*P*						0.043^∗^	0.038^∗^

Compared with the anlotinib group, ^∗^*P* < 0.05.

**Table 3:** The incidence of adverse reactions in 2 groups was compared (*n*(%)).

Adverse reactions	Anlotinib (*n* = 17)	Combination (*n* = 26)	*P*
Hypertension	5 (29.41)	10 (38.46)	0.045^∗^
Proteinuria	2 (11.76)	12 (46.15)	0.032^∗^
Rash	5 (29.41)	7 (26.92)	0.638
Nausea and vomiting	3 (17.64)	10 (38.46)	0.043^∗^
Leukopenia	1 (5.88)	3 (11.54)	0.829
Transaminase goes up	3 (17.65)	5 (19.23)	0.762
Creatinine increased	1 (5.88)	6 (23.08)	0.028^∗^

Compared with the anlotinib group, ^∗^*P* < 0.05.

## Data Availability

The data that support the findings of this study are available on request from the corresponding author. The data are not publicly available because they contain information that could compromise research participant privacy.

## References

[1] Bray F., Ferlay J., Soerjomataram I., Siegel R. L., Torre L. A., Jemal A. (2018). Global cancer statistics 2018: GLOBOCAN estimates of incidence and mortality worldwide for 36 cancers in 185 countries. *CA: a Cancer Journal for Clinicians*.

[2] Schabath M. B., Cote M. L. (2019). Cancer progress and priorities: lung cancer. *Cancer Epidemiology, Biomarkers & Prevention*.

[3] Torre L. A., Siegel R. L., Jemal A. (2016). Lung cancer statistics. *Advances in Experimental Medicine and Biology*.

[4] Siegel R. L., Miller K. D., Jemal A. (2015). Cancer statistics, 2015. *CA: a Cancer Journal for Clinicians*.

[5] Collins L. G., Haines C., Perkel R., Enck R. E. (2007). Lung cancer: diagnosis and management. *American Family Physician*.

[6] Ai X., Guo X., Wang J. (2018). Targeted therapies for advanced non-small cell lung cancer. *Oncotarget*.

[7] Moya-Horno I., Viteri S., Karachaliou N., Rosell R. (2018). Combination of immunotherapy with targeted therapies in advanced non-small cell lung cancer (NSCLC). *Therapeutic Advances in Medical Oncology*.

[8] Nagano T., Tachihara M., Nishimura Y. (2019). Molecular mechanisms and targeted therapies including immunotherapy for non-small cell lung cancer. *Current Cancer Drug Targets*.

[9] Rolfo C., Caglevic C., Santarpia M. (2017). Immunotherapy in NSCLC: a promising and revolutionary weapon. *Advances in Experimental Medicine and Biology*.

[10] Imyanitov E. N., Iyevleva A. G., Levchenko E. V. (2021). Molecular testing and targeted therapy for non-small cell lung cancer: current status and perspectives. *Critical Reviews in Oncology/Hematology*.

[11] Solomon B. J., Mok T., Kim D. W. (2014). First-line crizotinib versus chemotherapy in ALK-positive lung cancer. *The New England Journal of Medicine*.

[12] Drilon A., Siena S., Ou S. I. (2017). Safety and antitumor activity of the multitargeted pan-TRK, ROS1, and ALK inhibitor entrectinib: combined results from two phase I trials (ALKA-372-001 and STARTRK-1). *Cancer Discovery*.

[13] Rotow J., Bivona T. G. (2017). Understanding and targeting resistance mechanisms in NSCLC. *Nature Reviews. Cancer*.

[14] Keller S., Schmidt M. H. H. (2017). EGFR and EGFRvIII promote angiogenesis and cell invasion in glioblastoma: combination therapies for an effective treatment. *International Journal of Molecular Sciences*.

[15] Yu X., Li W., Deng Q. (2017). Neoalbaconol inhibits angiogenesis and tumor growth by suppressing EGFR-mediated VEGF production. *Molecular Carcinogenesis*.

[16] Ahluwalia M. S., Becker K., Levy B. P. (2018). Epidermal growth factor receptor tyrosine kinase inhibitors for central nervous system metastases from nonlogmall cell lung cancer. *The Oncologist*.

[17] Shen G., Zheng F., Ren D. (2018). Anlotinib: a novel multi-targeting tyrosine kinase inhibitor in clinical development. *Journal of Hematology & Oncology*.

[18] Gao Y., Liu P., Shi R. (2020). Anlotinib as a molecular targeted therapy for tumors. *Oncology Letters*.

[19] Reck M., Shankar G., Lee A. (2020). Atezolizumab in combination with bevacizumab, paclitaxel and carboplatin for the first-line treatment of patients with metastatic non-squamous non-small cell lung cancer, including patients with EGFR mutations. *Expert Review of Respiratory Medicine*.

[20] Santos E. S. (2020). Treatment options after first-line immunotherapy in metastatic NSCLC. *Expert Review of Anticancer Therapy*.

[21] Maity S., Pai K. S. R., Nayak Y. (2020). Advances in targeting EGFR allosteric site as anti-NSCLC therapy to overcome the drug resistance. *Pharmacological Reports*.

[22] Zhu J., Li R., Tiselius E. (2017). Immunotherapy (excluding checkpoint inhibitors) for stage I to III non-small cell lung cancer treated with surgery or radiotherapy with curative intent. *Cochrane Database of Systematic Reviews*.

[23] Ruan X., Shi X., Dong Q. (2019). Antitumor effects of anlotinib in thyroid cancer. *Endocrine-Related Cancer*.

[24] Forman A., Sotelo J. (2020). Tumor-based genetic testing and familial cancer risk. *Cold Spring Harbor Perspectives in Medicine*.

[25] Fujioka N., Bitterman P. B. (2012). Molecular targeted therapy in lung cancer. *Minnesota Medicine*.

[26] Bernicker E. (2015). Biomarker testing in non-small cell lung cancer: a clinician's perspective. *Archives of Pathology & Laboratory Medicine*.

